The article "Mental Health Education for Primary School Teachers in Areas Lacking Environmental Resource Dilemma and Countermeasures" was retracted in 2023. Reasons: signs of a paper mill; suspected computer-generated content; unreliable results or conclusions; lack of ethics approval or compliance.

# Mental Health Education for Primary School Teachers in Areas Lacking Environmental Resource Dilemma and Countermeasures

**DOI:** 10.1155/2022/4542385

**Published:** 2022-09-16

**Authors:** Qiuge Wang

**Affiliations:** School of Teacher Education, Pingdingshan University, Pingdingshan 467000, China

## Abstract

With the development of society and the progress of education, primary school teachers in areas lacking in environmental resources were facing many problems, and teachers' mental health problems were facing many challenges. The primary education conditions in the areas lacking in environmental resources were limited, and the education level needs to be improved. Therefore, the primary school teachers in the areas lacking in environmental resources should keep a good psychological state and make greater contributions to the primary education in the areas lacking in environmental resources. As the leader of primary education activities, teachers had a direct and profound influence on the growth and development of pupils in the enlightenment stage. Therefore, it was necessary to change the education and teaching concept, move towards the mental health education concept in the areas with poor environmental resources, strengthen the training of teachers' mental health education literacy, and actively explore the new mode of teacher education.

## 1. Overview

The mental health status of primary school teachers in areas lacking environmental resources was very important, which was related to the level of primary education [1]. In order to make the environment resources area children access to quality education and the statistical data of primary school teachers' mental health in recent years, the survey was shown in Figure 1, based on the environmental resources in primary school teachers' mental health problems as a starting point, exploring the promotion environmental resources area elementary school teachers' psychological health status of the effective measures.

## 2. Theory and Method

### 2.1. Definition of Mental Health Education for Primary School Teachers

With the gradual promotion of in Chinese cultural education classroom teaching reform, teachers, as the direct participants and leaders of this reform and innovation, are more and more concerned about from all sectors of society [2]. In recent years, studies have shown that the mental health level of primary and secondary school teachers is worrying, with nearly 30 percent of teachers having minor mental health problems [2]. As shown in Figure 2 below, special attention is paid that, compared with middle school and high school teachers, primary school teachers are more likely to be in a state of extreme fatigue and completely lose their enthusiasm for work. They are negative and insensitive to their students' attitudes. Maybe the primary and secondary schools are very young. Therefore, primary and secondary schools should not only pay attention to the study of students' courses but also pay attention to their life. Therefore, it is of great practical significance to care about the mental health of primary school teachers and the harm to students' sustainable development [3]. This situation is particularly evident in primary school teachers in areas with insufficient resources in the natural environment system.

The article "Mental Health Education for Primary School Teachers in Areas Lacking Environmental Resource Dilemma and Countermeasures" was retracted in 2023. Reasons: signs of a paper mill; suspected computer-generated content; unreliable results or conclusions; lack of ethics approval or compliance.

Regarding the concept of teachers ‘mental health, different scholars give different types of standards and structures closely around teachers' mental health. The norms of teachers' mental health include the recognition of teachers' role, selfless dedication to the cause of education, love for the cause of education, have a correct understanding of yourself, creativity to educate, and, in educational activities and daily life, can properly control emotions. Some scholars believe that basic education teachers should have five mental health qualities: cognition, emotion, personal behavior and belief, personality, and ability. According to the above insights, the relevant definition of teachers' mental health can be expressed as follows. Teachers' mental health refers to a stable and positive attitude in classroom teaching and daily life, which is reflected in the love of education, care for students, clear self-identity and character cognition, active learning attitude, active working attitude, and active learning attitude. They stabilize emotions, proper personal behavior can maintain harmonious interpersonal communication, calmly deal with social development and changes, and maintain stability [4]. Teachers' mental health is the premise for teachers to shape lofty professional ethics and sound personality. On the other hand, it has a deep and lasting positive effect on students' health. Teachers' mental health level is an indispensable part of teacher management and is an important link of mental health education.

The cognitive view of teachers ‘mental health education refers to the most basic and understanding view of teachers' mental health education, which has the role of correct guidance, adjustment, correct guidance, and manipulation. The influence of teachers ‘cognitive awareness on mental health education depends on the most basic attitude and emotional mode of teachers to mental health education, which is related to the significance of mental health education and the realization of value and also related to the development trend of students' mental health.

The article "Mental Health Education for Primary School Teachers in Areas Lacking Environmental Resource Dilemma and Countermeasures" was retracted in 2023. Reasons: signs of a paper mill; suspected computer-generated content; unreliable results or conclusions; lack of ethics approval or compliance.

### 2.2. Factors Contributing to Mental Health Problems

Primary education standards are more difficult in areas with insufficient environmental system resources. Teachers rooted at the grass-roots level have made outstanding contributions to the rapid development of grass-roots education, and the quality and level of primary school education in areas with poor environmental resources have been improved. Primary school teachers in areas with poor environmental resources need to have a healthy psychology, so that in order to further improve the teaching level of primary schools in areas with poor environmental resources and to provide better education for students in areas with poor environmental resources. At present, the mental health status of primary school teachers in areas with scarce environmental resources is worrying. First, primary school teachers in areas with poor environmental resources are facing great educational mental pressure [5]. At present, the mental health status of primary school teachers in areas lacking of environmental resources was not optimistic. First of all, primary school teachers in areas lacking of environmental resources bear great psychological pressure of teaching. At present, primary school teachers in areas lacking environmental resources were in short supply, and many teachers have to undertake multisubject teaching tasks, which makes primary school teachers in areas lacking environmental resources have a huge workload. Second, primary school teachers in areas lacking environmental resources face “career bottleneck” [6]. Although the education department has clearly stipulated that professional title evaluation was more favorable to primary schools in areas with poor environmental resources, the preferential policy has not been fully implemented, and many teachers in areas with poor environmental resources do not have time to publish “teaching and research theses” due to work pressure, which makes them unable to move forward in the “professional title evaluation.” Finally, in areas with scarce environmental resources, teachers' sense of professional honor is weak to cope with the high expectations between parents and the actual differences in primary schools. Parents in the areas with poor environmental resources regard “child education” as the only way to solve the areas with poor environmental resources and place hope on the students' learning and education in fact. There is a relatively large gap in hardware configuration and teacher resources between primary and secondary schools in areas with insufficient environmental system resources and those with good environmental resources [7]. As shown in Figure 3 below, primary school teachers in areas with poor environmental resources cannot realize the “teacher sense of professional honor” in practical teaching, while primary school teachers in areas with poor environmental resources have relatively low classroom teaching initiative.

The article "Mental Health Education for Primary School Teachers in Areas Lacking Environmental Resource Dilemma and Countermeasures" was retracted in 2023. Reasons: signs of a paper mill; suspected computer-generated content; unreliable results or conclusions; lack of ethics approval or compliance.

### 2.3. Influence of Teachers' Mental Health on Students' Development

Primary school teachers, as the key figures in education activities, have a direct and profound impact on the growth of students in the enlightenment stage and subtly affect the development of pupils' mental health [8]. The importance of specific teachers' mental health in quality-oriented education was obvious, as shown in Figure 4.

#### 2.3.1. Impact on Students' Academic Development

The Rosenthal effect shows that teachers' expectations of students will affect students' attitudes and behavior in learning. In education, if teachers can maintain a positive and optimistic attitude, a stable and peaceful attitude, and an open attitude, they can give students more positive support and encouragement and play an extremely important role in promoting students' academic development. The physical and mental health of primary and secondary school teachers should build a more active, independent, and equal classroom teaching and learning atmosphere and support the development trend of students' compassion behavior by showing out a lot of diversity to students. Satisfy the pupils basic psychological needs, such as ability and ownership, stimulate students' active learning motivation, so as to guide the student to maintain a positive attitude to learning, strong interest and curiosity in learning, and willing to actively explore disciplinary knowledge and skills [9, 10]. Relevant survey data were as follows Table 1.

Teachers' personal charm is one of the main external factors of students' academic emotions also embodies the teachers' mental health is the main harm of students' academic emotional development have active personal psychological quality teachers can with the help of its cheerful and open emotion feeling pure students, make the students in the learning education activities and homework experience happy, peaceful active academic emotions [11]. Emotion is closely related to the development of cognitive ability processing level, which can arouse the learning potential of students ‘curriculum and promote the development of students' creativity and independent innovation ability. Conversely, if the teacher constantly expresses the denial of the emotions to the students, the students will fall into the negative academic emotions such as fear, shame, and boredom. For a long time, this mood is easy to cause mental health problems, not conducive to the healthy and happy growth of students. The influence of teachers' mental health on students' academic development is also reflected in students' learning behavior and study. According to the mentality of Sven Gran Eriksson (Sven Gran Eriksson) and the eight-link basic theory of social development, school-aged children are facing the arduous task of developing an inferiority complex. All kinds of daily tasks can be done completed, get a sense of hardship. This kind of fatigue is mainly manifested in the habit of learning and the participation of various activities. Mental health primary and secondary school teachers in the daily education and teaching work can mainly show the students' recognition and support, encourage the students to actively learning goals, and participate in various theme activities, showing excellent [12]. On the other hand, primary and secondary schools with poor mental attitude and mental health problems may not be able to give sufficient care to students, which will have a bad impact on students' curriculum learning and reduce their self-esteem.

The article "Mental Health Education for Primary School Teachers in Areas Lacking Environmental Resource Dilemma and Countermeasures" was retracted in 2023. Reasons: signs of a paper mill; suspected computer-generated content; unreliable results or conclusions; lack of ethics approval or compliance.

#### 2.3.2. Influence on Students' Personality Development

Compared with early childhood, primary school students' self-consciousness is obviously directly affected by external factors, and the establishment of self-awareness of social development is accelerated. Among them, the harm of teachers ‘mental health to the sustainable development of primary school students' self-awareness cannot be underestimated. Mental health teachers show a more positive side in the daily education work with primary school students, treat students with a fair and fair attitude, attach importance to students' autonomy and uniqueness, and assist primary school students to create an objective and comprehensive self-consciousness and an independent and relatively stable personal evaluation management system. [13]. At this time, as long as you can give every student full respect and love, you can help the students to develop from low to high through the inside-out identity. In the development of self of primary school self-awareness, one of the trend factors that need to be paid attention to is the rapid development of self-esteem. Children's self-esteem is an emotional experience, and children's self-emotional experience developed to a higher level will produce self-esteem. Children with high self-esteem have a higher ability and sense of value and often maintain their own active cognitive ability and evaluation. Children with low self-esteem will feel inadequate, feel helpless, reduce their sense of self-worth, question themselves, or give up their [14], as shown in Figure 5 below. Therefore, the primary school teachers always maintain an active will quality and let the students experience the full support and respect of the teachers, to create a high degree of self-esteem. Ignoring the existence of students' self-consciousness, who endlessly release negative emotions for students, will damage students' self-esteem, so that students' ability and sense of value greatly reduced.

The article "Mental Health Education for Primary School Teachers in Areas Lacking Environmental Resource Dilemma and Countermeasures" was retracted in 2023. Reasons: signs of a paper mill; suspected computer-generated content; unreliable results or conclusions; lack of ethics approval or compliance.

As a key link in the construction of primary school students' personality, teachers and parents must pay attention to find the personality problems common to primary school students as soon as possible and take measures to solve [15]. Scholars have summarized the more common personality problems in modern primary school students from the five dimensions of self-regulation, IQ, social ideology, introversion, and emotion. The typical problems are the long-term use of electronic devices, slowly swallowing, unable to focus on learning and training, love angry, etc. Teachers' problem behavior is the external manifestation of mental health problems. Teachers' bad behavior and problem behavior usually give students psychological harm and psychological behavior problems derived from teachers. Data survey report, language violence in primary, and secondary school teachers often occur, and language violence is often accompanied by insulting language expression. Teachers will use insulting and discriminatory language expressions such as contempt and ridicule to students, which will make students cause inferiority complex, fear and other depression psychology, but their personality and self-esteem will also be infringed upon and harm. However, the primary and secondary school teachers with relatively high mental health level harm the students because of their passion, kindness, independent, and honest personality style and help them to create a sound personality.

#### 2.3.3. Influence on Students' Social Development

In terms of teacher-student relationship, the teacher-student relationship of primary school students has the characteristics of intimacy, responsiveness, and conflict, which reflect that teachers and students will not only have positive interpersonal interaction but also may appear conflict between teachers and students. In the heart of love and responsibility of teachers and students to establish a democratic, equal, harmonious, and intimate relationship between teachers and students, teachers and students can cooperate with each other, common cooperation, mutual tolerance, and understanding. If the teacher has no love in his heart and only overrules the students with cold commanding authority, he will be resisted by the students, resulting in contradictions and conflicts. In addition, teachers' partiality towards some students will also lead to problems in the teacher-student relationship and affect students' views on interpersonal communication and the cultivation of their skills [16].

The article "Mental Health Education for Primary School Teachers in Areas Lacking Environmental Resource Dilemma and Countermeasures" was retracted in 2023. Reasons: signs of a paper mill; suspected computer-generated content; unreliable results or conclusions; lack of ethics approval or compliance.

In the peer relationship, the establishment of friendship and peer generation is the main characteristics of primary and secondary schools to get along with people. Physical and mental health of primary school teachers in interpersonal communication also play a certain leading role in the rapid development of primary school students' peer association. If teachers can respect, treat others equally and fairly in their daily work, and often give encouragement, support, and care for students, they can influence students imperceptibly, and students can help each other, get along harmoniously with their classmates, and create close friendship. If the teachers show the axial force, isolation, and discrimination in their daily work, and if they compete with their colleagues maliciously, the students will also be affected, for example, quarrel with friends and isolate others for compensation.

Today's rate of social change is beyond imagination, and emergencies such as COVID-19 encourage people to think about the importance of social adaptability in personal career development. Primary school students are also beginning to encounter more and more social and life variability, including the transformation of peers, different types of social roles, and various kinds of extracurricular leisure activities. In order to calmly cope with social development trend and keep good social integration, primary school teachers guide students to accept their lover, promote his social personal behavior, shape students give full play to different types of social effect, objective understanding, and evaluation of the association between learning and entertainment, make students gradually self-knowledge and society in turn, primary and secondary schools ignore the students' curiosity about social daily life and exploration spirit, the students' course learning as a single criterion. Too much induction blocks the rapid development of students ‘social adaptability, resulting in students' depression and closure, avoidance, negative attitude, resistance, and other social integration problems.

#### 2.3.4. Influence on Students' Career Development

Today's educational reform has promoted the remodeling and reconstruction of the role of teachers, and traditional teachers have been endowed with new roles and positioning, and one of the important trends of transformation includes the transformation from “professional training instructor” to “guide of students' life development.” With the implementation of online education and other technologies, the main task of teachers will return from “teaching” to “educating,” putting more time and energy on the exploration and planning of each student's psychological growth and career development, actively exploring students' positive psychological quality and potential, and giving students more personalized guidance. Teachers with an open and inclusive attitude to the development of the times can actively adapt to the pace of the times and social development, actively pay attention to the latest career development trends in various fields, help primary school students understand and contact with different professions and their necessary conditions and skills, and guide primary school students to establish a correct career outlook and outlook on life. Gradually cultivate primary school students' awareness and ability of career exploration and career planning [17].

The article "Mental Health Education for Primary School Teachers in Areas Lacking Environmental Resource Dilemma and Countermeasures" was retracted in 2023. Reasons: signs of a paper mill; suspected computer-generated content; unreliable results or conclusions; lack of ethics approval or compliance.

### 2.4. Countermeasures to Improve Mental Health

#### 2.4.1. Government Department Education Departments Should Give Priority in Policy

The most critical countermeasure to improve the mental health of primary school teachers in areas lacking environmental resources is the high attention of the government. It is necessary for the government and relevant education departments to increase the policy preference and allocation of funds to reduce the number of teachers in areas with poor environmental resources, enhance the title of primary school teachers, and develop areas with poor environmental resources and their promotion space. On the other hand, the government departments should increase the financial input in education in areas lacking environmental resources. In the case of sufficient funds, primary schools in areas with scarce environmental resources can attract “high-paying positions,” expand the team of primary school teachers in areas with scarce environmental resources, and alleviate the task volume of teachers. For example, the education department can invest part of the education in primary school teaching in areas with special environmental resources shortage, promote the development trend of primary school education in areas with environmental resources shortage, get sufficient funds, attract more teachers, and expand the primary school teachers in areas with environmental resources shortage. On the other hand, the education departments of the government departments should increase the preferential policies for the primary education in the areas with scarce environmental resources. For example, to ensure the work and life of rural primary school teachers, the current policies on professional job appraisal and performance reward should be formulated to make the salary and performance appraisal salary of primary school teachers in areas with poor environment and resources safer. This can motivate primary school teachers in resource-poor areas.

The article "Mental Health Education for Primary School Teachers in Areas Lacking Environmental Resource Dilemma and Countermeasures" was retracted in 2023. Reasons: signs of a paper mill; suspected computer-generated content; unreliable results or conclusions; lack of ethics approval or compliance.

#### 2.4.2. Rich and Colorful Entertainment Life Methods of Teachers

The cities where primary schools are located in areas with environmental resources are generally far away from the urban areas, which brings great inconvenience to the living conditions of primary school teachers in areas with shortage of environmental resources. In areas with a shortage of environmental resources, many primary and secondary schools have settled down for many years, with few leisure activities and lack of normal communication with people. This kind of working growth environment does not benefit from the mental health of primary school teachers in areas with poor environmental resources. Because of such things, give entertainment programs for teachers. In the library, computer laboratory, badminton venues, and other places can create small classrooms, for teachers to give leisure and entertainment clubs. After a busy day of work, exercise and reading can relax. As primary school teachers in environmental and resource areas, they should maintain a stable working attitude and assist teachers to produce healthy psychological [18]. In addition, teachers should also promote interpersonal communication. For example, we can create some research institutes, organize some leisure activities during vacation institutions, and give us opportunities to communicate with each other. The theme activity will communicate with colleagues and like-minded friends about their work experience, share the interest in life, and reduce the “thick” psychological state in teacher education. Better and effective communication can also build a harmonious working environment, so that teachers can maintain a happy mood in the work and maintain a friendly and equal attitude towards students.

#### 2.4.3. Make Full Use of Initiative

As primary school teachers in areas with scarce environmental resources, we should fully understand the necessity of maintaining the “physical and mental health and mental outlook,” which is also the most basic professional requirement of teachers. Therefore, primary school teachers in areas with scarce environmental resources must make full use of their initiative to maintain a healthy mental state. First, they should face the work pressure properly. In the face of heavy teaching content, teachers must maintain an active psychological state and properly face the current situation, according to the scientific and reasonable planning and systematic teaching content. Second, to stimulate the potential. Primary school teachers in areas with weak environment and resources should resist the temptation, strengthen ideological education and learning, diligently shape their personality traits, and constantly improve the level of moral education. For example, if other teachers have their own efficacy and welfare protection, the primary school teachers in areas with scarce environmental resources need to fully realize their own shortcomings, curb their wrong ideas, and remain optimistic. Third, be active and gain educational ability. Primary school teachers in resource-poor areas should always be student-oriented and learn advanced educational ideas, ideas and professional knowledge, and their own cultural and educational abilities, so as to provide students with better educational services.

The article "Mental Health Education for Primary School Teachers in Areas Lacking Environmental Resource Dilemma and Countermeasures" was retracted in 2023. Reasons: signs of a paper mill; suspected computer-generated content; unreliable results or conclusions; lack of ethics approval or compliance.

## 3. Solutions and Strategies

### 3.1. Mental Health Care about Mental Health Level

Personally, I think the most direct and effective way to improve and maintain the mental health of primary school teachers is self-adjustment. Learning innovative basic knowledge of mental health, understanding the way of mental attitude adjustment, and grasping the most basic knowledge and skills of mental health can promote and maintain their own mental health level. At the same time, primary school teachers can also create an active will quality in their daily work and life, including a high sense of responsibility, tolerance for children, moral quality, vitality, attention, keen observation, and emotional control ability. Therefore, the efficient mental health and mental health culture education ability [19] is as shown in Figure 6 below.

From the school level, the school should actively build a beautiful campus, create a beautiful campus natural environment, and at the same time provide a relaxed and supportive interpersonal environment and humanistic care, so that primary school teachers can obtain a sense of security and satisfaction in the school environment. In addition, when organizing vocational training for primary school teachers, schools should increase the training content of mental health education and help primary school teachers to master the knowledge and strategies of mental health education in a more systematic and scientific way through a training system with clear objectives, detailed contents, scientific methods, and modern means, as shown in Table 2.

On the social level, compared with other professional groups, primary school teachers have contradictory social and economic status, that is, teachers' high social expectations and their real salary have a significant gap. Therefore, all sectors of society should sort out the expectations of primary school teachers and give sufficient understanding and support. At the same time, the government should increase investment in education; strive for primary school teachers' salaries, housing, medical treatment, and other material treatment; formulate preferential policies; constantly improve the working and living standards of primary school teachers; improve their employee satisfaction; and reduce the probability of mental health problems. With the big data technology of primary and secondary school teachers in China as the carrier, the psychological education mode of primary and secondary school teachers includes five elements of objective diagnosis, data collection, data statistical analysis, management decision-making, and monitoring and early warning information, which can support and guarantee teachers' mental health and immediately monitor their mental health problems.

The article "Mental Health Education for Primary School Teachers in Areas Lacking Environmental Resource Dilemma and Countermeasures" was retracted in 2023. Reasons: signs of a paper mill; suspected computer-generated content; unreliable results or conclusions; lack of ethics approval or compliance.

### 3.2. Focus on Specific Problems and Further Explore the Influencing Mechanism

Mental health of primary school teachers is the definition of mental health in special professional fields, and mental health is very broad. To explore the mental health of primary school teachers and the impact on students' growth, we must classify and discuss the research content, research methods, and research objects more thoroughly.

The research content needs to pay attention to more specific mental health problems of primary school teachers, including the current situation and cause of teachers' softness, teachers' work pressure, and teachers' job burnout and the influence mechanism on students' sustainable development.

In terms of research methods, we can adopt the most widely used investigation and research method, and personal evaluation can also be closely combined with other comments, tracking scientific research, interviews, and other research methods, so as to analyze the specific problems of mental health of primary school teachers from various aspects. For example, the most typical trial paradigm, such as Stroop task, Oddball paradigm, and Go-Nogo paradigm, as shown in Table 3, is used to expand the basic idea.

For the research objects, primary school teachers can be screened from different perspectives to discuss different specific mental health problems of primary school teachers. It is divided into female teachers and male teachers according to gender. According to the job responsibilities, it can be divided into primary school teachers, different curriculum teachers, and primary school teachers [20]. According to each stage of the development of teachers' technical majors, teachers are divided into special groups such as preworking teachers, beginner teachers, and authoritative expert teachers, so as to get the main differences, problems, and influences of the mental health of primary and secondary school teachers in different special groups.

The article "Mental Health Education for Primary School Teachers in Areas Lacking Environmental Resource Dilemma and Countermeasures" was retracted in 2023. Reasons: signs of a paper mill; suspected computer-generated content; unreliable results or conclusions; lack of ethics approval or compliance.

### 3.3. Get Rid of the Negative Effects and Play a Positive Effect

The mental health of primary school teachers is related to the development of students in all aspects. Primary school teachers in the emotion, personality, personal behavior, and other aspects of the performance that are not very good will have a bad impact on the development of students. Primary school teachers should be good at maintaining active, stable mental health, optimistic to others, and perfect personality. They will subtly harm students' learning feelings, friendly interpersonal behavior, and the active promotion of environmental factors. Therefore, primary school teachers should attach great importance to their own mental health and the impact on students' development, get rid of the bad impact of poor mental health problems on students' development and mental health level, make full use of the positive role in their student development, and promote students' physical health and sustainability of below [21], as shown in Figure 7.

## 4. Conclusion

In short, healthy psychology is the premise to improve the teaching level of primary school teachers in areas where environmental resources are scarce [22]. Teachers have a healthy psychology, which is conducive to cultivating students' positive mentality and effectively helping students establish a correct world outlook, outlook on life, and values. Therefore, society, government, schools, and teachers should form an educational joint force to work together to cultivate the healthy psychology of primary school teachers in areas where environmental resources are scarce. As the leader of primary education activities, teachers have a direct and profound impact on the growth and development of primary school students who are in the stage of enlightenment. Therefore, we should change the concept of education and teaching, move towards the concept of mental health education in areas where environmental resources are scarce, strengthen the training of teachers' mental health education literacy, and actively explore new models of teacher education.

## Figures and Tables

**Figure 1:** Research on the demand for mental health education.

**Figure 2:** Mental health distribution of teachers.

**Figure 3:** Causes of mental health of teachers.

**Figure 4:** The importance of mental health in quality education.

**Figure 5:** Influence of mental health on personality development.

The article "Mental Health Education for Primary School Teachers in Areas Lacking Environmental Resource Dilemma and Countermeasures" was retracted in 2023. Reasons: signs of a paper mill; suspected computer-generated content; unreliable results or conclusions; lack of ethics approval or compliance.

**Figure 6:** Three-dimensional structure of health.

**Figure 7:** Several aspects of positive effects of mental health.

**Table 1:** Psychological health survey of students.

Title	Not	Sometimes	From time to time	Often	Always
1. No extracurricular activities	1	2	3	4	5
2. Mood was up and down	1	2	3	4	5
3. Cross-check operation	1	2	3	4	5
4. I think people do not like me	1	2	3	4	5
5. Feel depressed	1	2	3	4	5
6. Nervous	1	2	3	4	5
7. Lack of motivation	1	2	3	4	5
8. Not fit in with school life	1	2	3	4	5
9. I feel the social atmosphere was not good	1	2	3	4	5
10. Do things slowly	1	2	3	4	5
11. Think differently	1	2	3	4	5
12. Worry about untidy clothes	1	2	3	4	5
13. Easy to cry	1	2	3	4	5
14. Feel hopeless about your future	1	2	3	4	5

**Table 2:** Statistical table of mental health education and training.

The serial number	The training content	Class number	The speaker
1	Introduction to school mental health education	10 hours	
2	Adolescent developmental psychology	20 hours	
3	Educational psychology	15 hours	
4	Mental hygiene	30 hours	
5	Curriculum design and implementation	25 hours	
6	Teacher mental health and health care	10 hours	
7	Methods to deal with students' psychological problems	20 hours	

**Table 3:** Mental health teachers in higher vocational colleges in Yunnan province participated in the project in recent three years.

	Number	Percentage		Frequency	Percentage
Never take part in	12	28.57	Field project	39	50.00
One or three times	22	52.38	The municipal project	21	26.92
More than 3 times	8	19.05	Provincial subject	18	23.08
			National subject	0	0
Total	42	100	Total	78	100

## Data Availability

The labeled data set used to support the findings of this study is available from the corresponding author upon request.

## References

[1] Kerebih H., Abrha H., Frank R., Abera M. (2018). Perception of primary school teachers to school children’s mental health problems in Southwest Ethiopia. *International journal of adolescent medicine and health*.

[2] Prabhu V., Ashok L., Kamath V. G., Kamath A., Chandrasekaran V. (2019). Exploring Teachers Perspectives on Mental Health Disorders-A Preliminary Study. *Indian Journal of Public Health Research & Development*.

[3] Granrud M. D., Anderzèn‐Carlsson A., Bisholt B., Steffenak A. K. (2019). Public health nurses’ perceptions of interprofessional collaboration related to adolescents’ mental health problems in secondary schools: A phenomenographic study. *Journal of Clinical Nursing*.

[4] Anderson M., Werner-Seidler A., King C., Gayed A., Harvey S. B., O’Dea B. (2019). Mental health training programs for secondary school teachers: a systematic review. *Journal of School Mental Health*.

The article "Mental Health Education for Primary School Teachers in Areas Lacking Environmental Resource Dilemma and Countermeasures" was retracted in 2023. Reasons: signs of a paper mill; suspected computer-generated content; unreliable results or conclusions; lack of ethics approval or compliance.

[5] Egan T. E., Wymbs F. A., Owens J. S., Evans S. W., Hustus C., Allan D. M. (2019). Elementary school teachers’ preferences for school-based interventions for students with emotional and behavioral problems. *Psychology in the Schools*.

[6] Otten J. J., Bradford V. A., Stover B. (2017). The culture of health in early care and education: a comparative study on the health of workers in China. *Journal of Health Science And Technology*.

[7] Mathews F., Newlove-Delgado T., Finning K. (2019). Teachers’ concerns about pupil’s mental health in a cross-sectional survey of a population sample of British schoolchildren’s hope for a healthy future. *Schoolchildren’s Hope for a healthy future*.

[8] Huang Y. H., Ling P., Lin Y., Wong R., Lee M., Wong M. (2021). Teachers’ attitude and feelings of self-efficacy toward student mental health needs. *American Journal of Occupational Therapy*.

[9] Le T. P., Hsu T., Raposa E. B. (2021). Effects of natural mentoring relationships on college students’ mental health: the role of emotion regulation. *American Journal of Community Psychology*.

[10] Reyes C. R., Gilliam W. S. (2021). Addressing challenging behaviors in challenging environments: findings from Ohio’s early childhood mental health consultation system. *Development and Psychopathology*.

[11] Dhapani V. R., Chrasekaran S., Singh S., Sood M., Singh S. P. (2018). Community stakeholders’ perspectives on youth mental health in India: problems and recommendations in psychiatry. *Journal of Psychiatry*.

[12] Kankaanranta M., Mehtälä S., Hankala M., Merjovaara O., Rousi R. (2021). Children’s conceptions of mental well-being and ideas for its promotion through digital environments. *International Journal of Child-Computer Interaction*.

[13] Wells A. E., Hunnikin L. M., Ash D. P., van Goozen S. H. M. (2021). Improving emotion recognition is associated with subsequent mental health and well-being in children with severe behavioural problems. *European Child & Adolescent Psychiatry*.

[14] Ormiston H. E., Nygaard M. A., Heck O. C. (2021). Educator perspectives on mental health resources and practices in their school. *Psychology in the Schools*.

[15] Alakrash H. M., Razak N. A. (2021). Education and the fourth industrial revolution: Lessons from COVID-19. *Journal of Computers & Continua*.

[16] Ohrt J. H., Deaton J. D., Linich K., Guest J. D., Wymer B., Sandonato B. (2018). Teacher training in K-12 student mental health: systematic review. *Journal of Psychology in China*.

[17] Glazzard J., Rose A. (2020). The impact of teacher well-being and mental health on pupil progress in primary schools. *Journal of Public getting health*.

[18] Akihiro N., Machi K., Ryo H. (2020). Compulsory educational mental health support system in Japan. *Journal of Pediatrics international*.

The article "Mental Health Education for Primary School Teachers in Areas Lacking Environmental Resource Dilemma and Countermeasures" was retracted in 2023. Reasons: signs of a paper mill; suspected computer-generated content; unreliable results or conclusions; lack of ethics approval or compliance.

[19] Punukollu M., Leighton E. L., Brooks A. F. (2020). SafeSpot: an innovative app and mental health support package for Scottish schools – a qualitative analysis as part of a mixed methods study. *Child and adolescent mental health*.

[20] Patra S., Patro B. K. (2020). COVID-19 and adolescent mental health in India. *The Lancet Psychiatry*.

[21] Hou J. (2022). Effective ways for college students’ mental health education based on music therapy. *Journal of Healthcare Engineering*.

[22] Jin Y. (2022). The promoting effect of mental health education on students’ social adaptability: implications for environmental. *Journal of Environmental and Public Health*.

